# Multiresponse Optimization of Linkage Parameters of a Compliant Mechanism Using Hybrid Genetic Algorithm-Based Swarm Intelligence

**DOI:** 10.1155/2021/4471995

**Published:** 2021-12-24

**Authors:** Rami Alfattani, Mohammed Yunus, Turki Alamro, Ibrahim A. Alnaser

**Affiliations:** ^1^Department of Mechanical Engineering, College of Engineering and Islamic Architecture, Umm Al Qura University, Mecca, Saudi Arabia; ^2^Department of Mechanical Engineering, King Saud University, Riyadh 11421, Saudi Arabia

## Abstract

This research focuses on the synthesis of linkage parameters for a bistable compliant system (BSCS) to be widely implemented within space applications. Initially, BSCS was theoretically modeled as a crank-slider mechanism, utilizing pseudo-rigid-body model (PRBM) on stiffness coefficient (*v),* with a maximum vertical footprint (*b*_max_) for enhancing vibration characteristics. Correlations for mechanism linkage parameters (MLPs) and responses (*v and b*_max_) were set up by utilizing analysis of variance for response surface (RSM) technique. RSM evaluated the impact of MLPs at individual/interacting levels on responses. Consequently, a hybrid genetic algorithm-based particle swarm/flock optimization (GA-PSO) technique was employed and optimized at multiple levels for assessing ideal MLP combinations, in order to minimize characteristics (10% *v* + 90% of *b*_max_). Finally, GA-PSO estimated the most appropriate Pareto-frontal optimum solutions (PFOS) from nondominance set and crowd/flocking space approaches. The resulting PFOS from validation trials demonstrated significant improvement in responses. The adapted GA-PSO algorithm was executed with ease, extending the convergence period (through GA) and exhibiting a good diversity of objectives, allowing the development of large-scale statistics for all MLP permutations as optimal solutions. A vast set of optimal solutions can be used as a reference manual for mechanism developers.

## 1. Introduction

This study presented a bistable compliant mechanism (BCM) concept design, together with an optimization method, based on selected output parameters. Synthesis of compliant mechanism design models can be presented in a myriad of formats, though all lead to the final necessary parameters for the individual mechanism dimensions. BCM aims to operate as a deployable unit cell, requiring one degree of freedom (i.e., one actuation input), and occurs within multiple applications such as developing structures, self-closing, gates, and switches [1, 2]. Such unit cells can be tessellated and arranged to execute shape-morphing systems in an organized pattern [3, 4] for morphing structures, increasing the ability to morph the unit cell surface profile when actuated, deploying space antennas, and aircraft wing flaps [5–7]. Should such designs be produced at microscale levels, they could be deployed within relays and medical grips [8]. The BCM can also be employed within automotive industries, in particular, as bumper collision absorber units and vehicular rear trunk lids [9].

The BCM mobility characteristic is obtained from flexible segment deflections, thus eliminating the requirement for mechanical joints, such that both output and costs are affected. The mechanism has moving parts, most of which are thin, with such sections being the first to bend whenever a force is applied or during displacement. There are two types of compliant mechanisms (CMs), partially or fully compliant. Full CMs can be mobilized without having any kinematic pairs. However, one or more joints (such as pins and sliders) are present within partial CMs, having the advantage of reduced friction, weight, and maintenance and improved reliability [1]. Furthermore, minimizing production time affects costs, since there are no hinges in its design, resulting in reduced component assembly workloads. CM accuracy is enhanced, since there are no pinpoint-induced vibrations, and force-induced vibrations are decreased [10, 11], rendering them highly attractive for employment within high-precision instruments [12]. The compliant-based hinges are also used in commercial articles like robots.

Moreover, a design can have the most efficient method for achieving mechanically stable robotic designs through CM incorporation [13, 14]. However, when using such a compliant process, there are certain challenges and limitations. If the compliant section is exposed to an extreme stress/temperature environment for extended periods, deformation issues can gradually manifest themselves [15]. Remaining within an elastic material range is challenging when the mechanism is deformed, as mobile segments are often employed for energy storage, thus imposing design limitations [16]. Consequently, researchers have developed approaches to model-compliant mechanisms for approximation.

The elliptic integral method is commonly used to solve large-deflection issues of compliant beams with loading conditions [17]. However, a closed-form solution for compliant loading condition mechanisms is challenging to derive, while approximation methods, such as pseudo-rigid-body models (PRBMs), are more useful, specifically in CM designing processes [18, 19]. PRBM is an approach for CM generation [1]. To discuss more insights, this study employs PRBMs. This approach can achieve topology optimization and obtain a nonlinear CM with assigned input/output parameters as an alternative implementation strategy [20, 21]. Su also applied polynomial homotopy to construct CM kinematic equations for solving targeted design outputs [22]. An approach involving a CM kit was conducted by Limaye, associating the characteristic from topology optimization, and this enables the development of a designed mechanism [23].

BCM elements were generated using the PRBM methodology, which was initially developed by Howell and Midha [1]. The PRBM is noncomplex and is employed for determining/identifying nonlinear beam activity with deflections. Depending on the beam's loading conditions, this method allows approximations of the flexural beam, using torsional springs to combine two (or more) rigid links. PRBM parameters include rigid link length, coefficient of stiffness, and torsional spring location. Such parameters explain the nonlinearity, together with the kinematic and force-deflection study for the mechanical system. To produce flexural section behavior, the compliant theory was employed for creating varying PRBM formats.

As in every design, an optimum solution is required for producing effective functionality. The design synthesis of the individual PRBM does not regulate structural error(s) at the precision points, though it is maintained within a set mobility range. To solve this problem, an optimization tool is important. The majority of previous literature treat fully compliant mechanisms as flexible continua, where it can be approached through methods such as size, shape, and topology optimization, assuming the flexible continuum remains in the structural form [24, 25]. Moreover, optimizing the nonlinear equation is too complex, which leads to the implementation of numerical optimization algorithms.

The parameter-regulating issue is critical within a genetic algorithm's performance, achieved by a self-adaptive approach (SAP), and based on entropy/nature rules for regulating algorithmic parameters. This approach utilizes entropy from both the population and each genetic locus as the feedback for evaluating the algorithmic status. Consequently, parameters are adjusted according to the algorithmic status and rules of nature. This strategy avoids the impact of randomness when evaluating algorithmic status and tracks the development of each gene in a timely manner, in order to prevent premature and nonconvergence on a specific gene. Furthermore, this method maintains solutions with decent quality, though also increases the probability that the solutions with poor quality could vary. Experimental results demonstrate that the proposed parameter-controlling strategy is valid for the algorithm to enhance problem-solving performance for solving multiple combinatorial optimization challenges [26].

In order to solve attribute selection issues for https://www.sciencedirect.com/topics/computer-science/classificationimproving grouping precisely, together with lowering computation difficulty, the data groups requiring processing by multiple classifiers within large-sized challenges must be analyzed. Such efficient problem-solving requires a self-adaptive parameter and a strategy-based PSO (SPSPSO) algorithm, which was proposed for GA-based systems, and has increased classifiers. SPSPSO can adjust both one candidate solution generation, with parameter values having good global and local search ability through four classifiers (*k*-nearest neighbor (KNN), linear discriminant analysis (LDA), extreme learning machine (ELM), and support vector machine (SVM)). These are individually utilized as evaluation functions for assessing effectiveness within SPSPSO-generated feature subsets. Experimental results demonstrate that SPSPSO improved GA performance. In addition, feature selection can improve classification accuracy and reduce computational timings for multiple classifiers. Furthermore, KNN is an improved surrogate model in comparison to other classifiers used in such studies [27].

Research findings are scarce, regarding multiresponse optimization in seeking the multiple combinatory MLP permutations for generating considerable quantities of optimized data and for ultimately producing a reference manual (required by designers/engineers) encompassing all possible response conditions. PSO methodology appears suitable for developing big data for the above requirement, while the other optimizing techniques could produce only one set of MLP combinations. Conversely, PSO provides Pareto-frontal optimized solutions, and selecting an optimized solution from these groups would be a challenging task. Likewise, GA can obtain optimized parameters. The hybrid method of combining GA with PSO techniques leads to rapid, more accurate results, nonrepetitive data, and cost effectiveness for multiresponse optimization in generating data for multiple MLP level combinations. Alternative methods, such as RSM [24], Taguchi [28], and fuzzy logic [14, 29], are unable to consider nonlinearities, with the resulting outcome accuracy being reduced, predicting only one set of MLP combinations for envisaging all possible output variations. GA techniques extend the convergence period in order to delve deeper into more accurate solutions produced by PSO techniques. Within our proposal, this study approaches the issue in two stages: initial PRBM development, followed by GA-PSO algorithm development as the optimum solution.

This study is implemented for two PRBM types: the fixed-pinned cantilever beam, which has a force at its end, and the initially curved pinned-pinned beam that utilizes torsional springs/flexural pivots having reduced length for their modeling. Other CM joints are flexural pivots of small lengths, having large displacement hinges with a motion range. Work is split into four stages as follows:

  Defining essential input and output variables for fixed-pinned cantilever beams and the initially curved pinned-pinned beam PRBM
  Generating mathematical models based on higher-order regression using ANOVA, with a recording of the most influential factors
  Using RSM Box–Behnken design with a desirable feature approach to carry out the multiobjective optimization to analyze various structural behaviors
  Using GA-PSO from MATLAB optimization toolbox, a vast possible-optimum combination of MLPs in achieving the minimum (90%) *b*_max_ and (10%) *ѵ* to develop a reference manual for engineers

## 2. Genetic Algorithm-Based Particle Swarm Optimization (GA-PSO)

GA-PSO is hybrid optimization, approximation, and systematic technique utilizing both swarm/flock intelligence to assess mechanism linkage parameters (MLPs) contributing to maximization/minimization state of fitting functions (FFs), combined with a genetic program that delays solution convergence. Typically, machine learning algorithms (namely, ANN and GA) are employed to combine optimum MLP values. Occasionally, algorithms demand the operator to allocate certain constants. Kennedy and Eberhart first demonstrated this in 1995, acquiring knowledge from bird/fish swarming patterns, focusing on evolution theory (similar to GA) [14, 29]. PSO has the capability to hold multiconceivable solutions simultaneously. It becomes very significant to maintain fitness for every solution gained from FF assessment, as each iteration is performed on each available particle within a fitness region (the latter achieves maximum FF through swarming/flying into it).

Response surface methodology (RSM) [24], Taguchi-based sensitivity analysis [25], hybrid Taguchi-differential evolution algorithm, and genetic algorithm [28, 30] refer to multiple other prevalent theoretical approaches for the synthesis of CMs in terms of shape optimization/topology. In order to simplify CM design using dimensional kinematic factors simultaneously, a two-stage approach is employed to analyze link dimensions with PRB diagrams and optimize flexure hinge dimensions using FEA results, through RSM. A multioutput optimization was also implemented to improve static/dynamic characteristics for the linear compliant guidance mechanism required by high-precision manufacturing processes. Through developing link kinematic associations, PRB diagram analysis and a mathematical model were developed using the analytical method to enhance the CM [31] synthesis method. In order to identify the optimum link dimensions for increasing design parameter quantities, gradient-based optimization was employed. FEA results from ADPL codes, within 3D structural model ANSYS, are used in RSM with the aid of assigned independent output variables. These factors have been transformed into mathematical models to determine optimal design variable sets.

The PSO method has disadvantages, such as difficulty in handling highly scattered issues, leading to poorly converged results within large iteration processes, and defined issues easily fall into high-dimensional space, which increases computational complexity [14]. PSO also requires large memory real estate and high processor speeds. GA implementation remains an art and a skill, as it requires less information on the issue while designing the objective function and obtaining the illustration and correct mathematical operator selection could be challenging. GA is also time-consuming [29].

## 3. Design Procedure

This section describes the model and the applied design procedures for a linear bistable compliant mechanism. In order to demonstrate the mechanism's bistable behavior, the tool will depend on the crank-slider mechanism and consider large deflection analysis. The kinetic/kinematic equations were numerically solved, derived from the PRBM. The representation allows for guideline generation design. Parameters employed in the design include the optimum force required to collect the actuator, material selection, compliant segment widths, optimum anticipated deflection, and optimum footmark. The latter includes examples such as the optimum rectangular region that fits the mechanism, and where the mechanism has free movement, without interfering with other components.

PRBM is an essential functional technique used to evaluate and synthesize a BCM. Howell and Midha first developed the approximations applied within the PRBM [31], by including identical behaviors between rigid body and CMs. The bistable compliant link 1 model is fixed-pinned PRBMs, with the link 2 model being the initially curved pinned-pinned beam, as shown in Figure 1. As a standardized method, virtual work was employed to derive the force-displacement equation for the compliant system. Concomitantly, Howell's constants were used as the PRBM constants, including the characteristic radius for the fixed-pinned *γ*, pinned-pinned *ρ*, and the rigidity coefficient KΘ, as shown in Table 1 [1, 3]. Illustrated in Figures 1(a) and 1(b), A, A′, and A″ are the first stable, unstable, and second stable configurations, together with related mechanism(s), respectively.

This section will divide the organization into three critical sections as follows:

  The theory underlies the BCM model, and a description will be given of how the model was derived from PRBMs.
  The step-by-step design would demonstrate design methods with dissimilar inputs.
  Steps for combining inputs and outputs using ANOVA, followed by RSM, are included in the derivation of quadratic-based regression models. Finally, steps for applying the Pareto front solver multiobjective PSO-based genetic algorithm will be demonstrated.

### 3.1. Modeling of Bistable Compliant Mechanism

The model's equations were obtained by solving the equations of kinetic and virtual work for an extended study [32]. The model sketches, parameters, and notations are shown in Figure 2. Determination of kinematic coefficient utilized kinematic equation. In order to form virtual work equations, the kinematic coefficient was consequently replaced. The model's equation was solved numerically and plotted.

(1) $$\begin{array}{c} L_{1}=l_{1}+l_{2}, \end{array}$$

(2) $$\begin{array}{c} l_{1}=\left(1-\gamma \right)L_{1},l_{2}=\gamma L_{1}. \end{array}$$

The mechanism gains its flexibility from the large deflection experienced by links 1 and 2 will buckles that also experience some deflection. Link 1 is split into two lengths *l*_1_ and *l*_2_.

Link 2 is split into three lengths *l*_3_, *l*_4_, and *l*_5_ on the basis of the pseudo-rigid body model, as shown in Figure 2.

(3) $$\begin{array}{c} L_{2}=l_{3}+l_{4}+l_{5}, \end{array}$$

(4) $$\begin{array}{c} l_{3}=l_{5}=\frac{\gamma L_{2}}{2},l_{4}=\left(1-\gamma \right)L_{2}. \end{array}$$

At the pseudo-rigid-body model of link 1, the characteristic stiffness *K*_1_ of the torsion spring is as follows:

(5) $$\begin{array}{c} K_{1}=\gamma K\Theta \frac{{\text{EI}}_{1}}{L_{1}},I_{1}=\frac{tw_{1}^{3}}{12}, \end{array}$$

(6) $$\begin{array}{c} K_{2}=\gamma K\Theta \frac{2{\text{EI}}_{2}}{L_{2}},I_{2}=\frac{tw_{2}^{3}}{12}, \end{array}$$

where *w* is the width of the link, *t* is the thickness of the link, and *E* is the material modulus of elasticity. The characteristic stiffness *K*_2_ is measured when linking two buckles. The moment equation can be calculated using *K*_2_ as follows:

(7) $$\begin{array}{c} M=\Theta_{1}K_{1}=F_{t}\gamma L_{1}, \end{array}$$

(8) $$\begin{array}{c} F_{t}=F_{B}\text{Sin}\left(\Theta_{1}+\theta_{1}+\theta_{2}\right), \end{array}$$

(9) $$\begin{array}{c} F_{B}\geq \pi^{2}E\frac{l_{2}}{L_{2}^{2}}. \end{array}$$

For simplification of design parameters, the equations are rendered nondimensional, as follows:

(10) $$\begin{array}{c} K\Theta \Theta_{1}=\frac{\pi^{2}}{2m\upsilon }\text{Sin}\left(\Theta_{1}+\theta_{1}+\theta_{2}\right), \end{array}$$

(11) $$\begin{array}{c} m=\frac{\sin\left(\theta_{1}\right)}{\sin\left(\theta_{2i}\right)}=\frac{L_{2}}{L_{1}}, \end{array}$$

(12) $$\begin{array}{c} \upsilon =\frac{K_{1}}{K_{2}}, \end{array}$$

where *F*_*t*_ and *F*_*B*_ are the internal forces of the links. For the mechanism, the near loop equations are as follows:

(13) $$\begin{array}{c} -x+l_{1}\cos\left(\theta_{1}\right)+l_{2}\cos\left(\theta_{1}+\Theta_{1}\right)+l_{3}\cos\left(\theta_{2}-\Theta_{2}\right)+l_{4}\cos\left(\theta_{2}\right)+l_{5}\sin\left(\theta_{2}+\Theta_{2}\right)=0, \end{array}$$

(14) $$\begin{array}{c} l_{1}\sin\left(\theta_{1}\right)+l_{2}\sin\left(\theta_{1}+\Theta_{1}\right)-l_{3}\sin\left(\theta_{2}-\Theta_{2}\right)-l_{4}\sin\left(\theta_{2}\right)-l_{5}\sin\left(\theta_{2}+\Theta_{2}\right)=0, \end{array}$$

where Θ_1_ is the link 1 PRBM angle, Θ_2_ is the link 1 PRBM angle, *θ*_2_ is the link 2 angle, and *θ*_1_ is the link angle 1. The virtual work equation was derived on the basis of the dependent variables (Θ_1_, Θ_2_, and *F*) and the specified independent variable (*x* and *θ*_2_) as follows:

(15) $$\begin{array}{c} \partial w=-F\text{d}x-\frac{\partial v}{\partial x}\text{d}x=0, \end{array}$$

(16) $$\begin{array}{c} F\frac{\partial x}{\partial \theta_{2}}\text{d}\theta_{2}-\frac{\partial v}{\partial \theta_{2}}\text{d}\theta_{2}=0, \end{array}$$

(17) $$\begin{array}{c} \frac{\partial v}{\partial x}=K_{1}\Theta_{1}\frac{\partial \Theta_{1}}{\partial x}+2K_{2}\Theta_{2}\frac{\partial \Theta_{2}}{\partial x}, \end{array}$$

(18) $$\begin{array}{c} \frac{\partial v}{\partial \theta_{2}}=K_{1}\Theta_{1}\frac{\partial \Theta_{1}}{\partial \theta_{2}}+2K_{2}\Theta_{2}\frac{\partial \Theta_{2}}{\partial \theta_{2}}, \end{array}$$

(19) $$\begin{array}{c} \frac{\partial \Theta_{1}}{\partial x}=\frac{\sin\left(\theta_{2}\right)}{l_{2}\cos\left(\theta_{1}+\Theta_{1}+\theta_{2}\right)}, \end{array}$$

(20) $$\begin{array}{c} \frac{\partial \Theta_{1}}{\partial \theta_{2}}=\frac{l_{4}+2l_{3}\cos\left(\Theta_{2}\right)}{l_{2}\cos\left(\theta_{1}+\Theta_{1}+\theta_{2}\right)}, \end{array}$$

(21) $$\begin{array}{c} \frac{\partial \Theta_{2}}{\partial x}=-\frac{\cos\left(\theta_{1}+\Theta_{1}\right)}{2l_{3}\sin\left(\Theta_{2}\right)\left[\cos\left(\theta_{1}+\Theta_{1}\right)\cos\left(\theta_{2}\right)-\sin\left(\theta_{1}+\Theta_{1}\right)\sin\left(\theta_{2}\right)\right]}, \end{array}$$

(22) $$\begin{array}{c} \frac{\partial \Theta_{2}}{\partial \theta_{2}}=\frac{l_{3}\sin\left(\theta_{1}+\Theta_{1}+\theta_{2}+\Theta_{2}\right)+l_{4}\sin\left(\theta_{1}+\Theta_{1}+\theta_{2}\right)+l_{5}\sin\left(\theta_{1}+\Theta_{1}+\theta_{2}+\Theta_{2}\right)}{l_{3}\left(\sin\left(\theta_{1}+\Theta_{1}-\Theta_{2}+\theta_{2}\right)-\sin\left(\theta_{1}+\Theta_{1}+\Theta_{2}+\theta_{2}\right)\right)}. \end{array}$$

The equations are derived to be nondimensional using these conditions, in order to enhance regulation of the design concept:

(23) $$\begin{array}{c} \zeta =\frac{F}{K_{1}}=F\frac{L_{1}^{2}}{K\Theta \gamma {\text{EI}}_{1}}. \end{array}$$

Equations (19)–(23) are used to form the nondimensional governing equation (16) to be numerically resolved:

(24) $$\begin{array}{c} \zeta +\Theta_{1}\frac{\partial \Theta_{1}}{\partial x}+2\frac{L_{1}}{\upsilon }\Theta_{2}\frac{\partial \Theta_{2}}{\partial x}=0, \end{array}$$

(25) $$\begin{array}{c} \Theta_{1}\frac{\partial \Theta_{1}}{\partial \theta_{2}}+2\frac{1}{\upsilon }\Theta_{2}\frac{\partial \Theta_{2}}{\partial \theta_{2}}=0. \end{array}$$

The solution of the governing equations (24) and (25) depends on the constant input parameters and the input variable parameters, as shown in Table 2 (*γ, K*Θ, and *E*).

For each input value set, numerical solutions will produce the values (*υ*, Θ_1_, Θ_2_, and *ζ*) as shown in Table 3. Using numerical solutions, the design outputs are obtained as follows:

(26) $$\begin{array}{c} L_{1}=\left(X-\frac{\Delta }{2}\right)\frac{1}{\cos\left(\theta_{1}\right)}, \end{array}$$

(27) $$\begin{array}{c} L_{2}=L_{1}\sqrt{{\left(\frac{\Delta }{2L_{1}}\right)}^{2}+\sin\;{\left(\theta_{1}\right)}^{2}}. \end{array}$$

The initial angle of link 2 (*θ*_2*i*_) can be calculated as follows:

(28) $$\begin{array}{c} \theta_{2i}=\;\cos^{-1}\left(\frac{\Delta }{2L_{2}}\right), \end{array}$$

(29) $$\begin{array}{c} w_{1}=\frac{\sigma y}{E}\frac{1}{\gamma K\Theta }\frac{L_{1}}{\Theta_{1}}, \end{array}$$

(30) $$\begin{array}{c} w_{2}=\sqrt[{3}]{\frac{m}{2\upsilon }}w_{1}, \end{array}$$

(31) $$\begin{array}{c} \beta =\frac{\zeta }{12{\left(\gamma K\Theta \right)}^{2}\Theta_{1}^{3}}=\frac{\gamma K\Theta {\text{EI}}_{1}\;\zeta }{L_{1}^{2}}, \end{array}$$

where *σ*_*y*_ is the yield stress of 35 MPa for the material selected (polypropylene) with Young's modulus (*E*) of 1.35 GPa. Regarding multiple sets of variable input parameters, the design outputs are solved numerically and presented in Table 3. The maximum linear deflection Δ and the maximum horizontal footmark *X* should be limited to satisfy the condition Δ ≤ *X*, ensuring that the mechanism complies with bistability geometric rules. Since they control the amount of force required to deform the mechanism between their two stable configurations, the concept of design relies on *υ* and *b*_max_. Consequently, in the following segment, these two outputs are optimized.

### 3.2. Multioutput Optimization Using GA-PSO Technique

Due to output requirements, such as minimizing both outputs *b*_max_ and *v*, obtaining more sets of an optimized parameter's combination becomes crucial, in order to validate all probable response variations. This was accomplished more accurately using mutation-based GA-PSO, rather than outdated approaches. FFs produce results whereby each output nominated for a particle existing in the fitness region has to be checked for its fitness. Such FF particles have maximum value, might swarm/fly into the fitness region and retain their position, individual best position, and velocity. The multiresponse optimization using PSO has dual goals: (1) convergence to the Pareto front for ideal global optimized solutions group and (b) supporting variation and scattering in solutions. Furthermore, the swarm/flock retained their global best position as well. PSO consists of the following six stages (refer to Figure 3):

The general aim of PSO with the GA process is to establish an unlimited group of Pareto front results or a pictorial subgroup. The nondominated (ND) solutions are results obtained by deteriorating one output and improving other outputs (and vice versa) to improve results while running a multioutput optimization. A Pareto front for best-global-optimized solutions group is achieved by strengthening the process within clashing outputs.

## 4. Results and Discussion

Numerous enhancing characteristics (*b*_max_ and *v*) for BSCS were subjected to optimization. Employing several approaches in the subsequent sections of its results enabled the MLPs combination to achieve responses (minimum of 90% *b*_max_ and 10% of *v*) for required conditions. Ultimately, an extensive set of improvised/optimized MLP data were revealed through the utilization of GA-PSO [29].

### 4.1. Data Fitness and Empirical Modeling for responses (considering ANOVA and R^2^)

Through applying Minitab^®^ software onto the outputs (*b*_max_ and v) and MLP data, as demonstrated in Table 3, empirical relations of high order (or quadratic level) were developed (refer to the following equations):

(32) $$\begin{array}{c} \upsilon =31.7+68*F-0.88*\Delta +0.58*X-0.25*\theta_{1}-5.2*t-10*F*F+0.0161*\Delta *\Delta +0.005*X*X-0.008*\theta_{1}*\theta_{1}-0.278*t*t-0.36*F*\Delta \\ +0.004*F*X-0.235*F*\theta_{1}-1.28*F*t-0.0384*\Delta *X+0.0358*\Delta *\theta_{1}+0.061*\Delta *t-0.0146*X*\theta_{1}+0.136*X*t-0.0178*\theta_{1}*t, \end{array}$$

(33) $$\begin{array}{c} b_{\max}=35.9-24.8*F-0.161*\Delta +1.042*X-3.155*\theta_{1}-0.48*t+6.59*F*F+0.0003*\Delta *\Delta -0.0196*X*X+0.03537*\theta_{1}*\theta_{1}+0.125*t*t-0.367*F*\Delta \\ +0.253*F*X+0.164*F*\theta_{1}-0.013*F*t+0.0165*\Delta *X-0.02202*\Delta *\theta_{1}-0.0016*\Delta *t+0.03954*X*\theta_{1}-0.0306*X*t+0.007*\theta_{1}*t. \end{array}$$

Fitness of empirical relation models was ERM-tested using ANOVA results of *b*_max_ and *v* (refer to Table 4), respectively, with MLPs' condition to be considered significant when *P*-value <0.05 and >*F*. Table 4 shows that as *P* is greater than *F*, developed ERMs proved to be very substantial models. In addition, the label *R*^2^ (square of multiple-regression coefficient), used as percentage model variability (from total variability), helps assure the noble relationship of developed ERM with theoretical analysis results [18]. ERM fitness is gauged by how closely the *R*^2^ value approaches 1. The *R*^2^ value was almost approaching 1 in the present work, confirming highly competent and adequate ERM results, when compared to the theoretical analysis. Table 4 shows that the degree/level of ERM resulted in good fitness relationships of 99 percent and 95 percent in contrast to theoretical data, with *R*^2^ values of 0.9982 for *b*_max_ and 0.9520 for *v*.

Consequently, both ERMs fulfill the fitness/competence/adequacy criteria.

### 4.2. Validation Experiments

ERMs obtained from the analysis of RS methodology for responses (*b*_max_ and *v*) were validated by comparing ERM predicted values corresponding to the theoretical results for the set of MLP levels available in Table 3, with a deviation of these results presented in Table 5. Deviations of ERMs predicted from theoretical results were found to be minute and lying in close (or better agreement) with the applied RS methodology (refer to Figure 4).

### 4.3. Impact of Individual and Interaction between MLPs on *b*_max_

In this segment, Pareto, factorial, and three-dimensional surface diagrams of two responses (*b*_max_ and *v*) were employed to valorize factor rankings (individually and in combinations). Out of five MLPs, *θ*_1_ (link 1 PRBM angle) is highly influential, followed by *X* and ∆ factors, detected from the Pareto diagram (given in Figure 5(a)). *θ*_*i*_, *X*, and ∆ were also observed, deciding MLPs in attaining theoretical *b*_max_. Normal distribution of data was found distributed in very close proximity to a line in Figure 5(b), indicating the ERMs' fit with the theoretical analysis used in Section 2.1. The individual MLPs at differing levels have an impact on *b*_max_, where *θ*_1_, the link 1 angle, is playing a more significant role, as the rotation of link 1 helps attain its maximum value. However, other MLPs such as *X* and ∆ also induce a degree of variation on *b*_max_. The MLPs *F* and *t* (the maximum force and link thickness) had minute/no effect on *b*_max_ with their level variation since other MLPs' variation hold *b*_max_ value easily (even with/without *F* and *t*). The type of effect (such as *X* > ∆ on *b*_max_) is also seen in Figure 6(a), which is the main requirement of these BCCS to assure that link 4 does not undergo buckling to retain the required link flexibility.

Combined or interactive impacting role(s) of MLPs on *b*_max_ (such as *F* and ∆; refer to Figures 6(b) and 6(c)) were observed in a manner that low/high *F*-value and ∆ reductions contributed to attaining *b*_max_. This condition is desired, as it helps maintain link stiffness and mechanism stability. Thus, *b*_max_ can be varied (higher or lower) by these two MLPs while maintaining all other MLPs at optimal values. Interactive impact levels for *F* and *X* on *b*_max_ are shown in Figures 6(b) and 6(d). Lowering *F* and increasing *X* would help attain optimal *b*_max._ Similarly, combining impacts of low *F*-values with increasing *θ*_1_ and *t* values would be significantly increasing *b*_max_ as shown in Figures 6(b), 6(e), and 6(f). These satisfy the condition of minimum value for maximum force *F*.

Referring to Figures 6(b), 6(g), 6(h), and 6(i), concerning the combined impact of minimum ∆ with increasing values of *X*, along with *θ*_1_ and *t* on *b*_max_, demonstrated how the maximum of it was achieved and satisfied the requirement of an ideal mechanism (i.e., *X* > ∆). Figures 6(b), 6(j), and 6(k) demonstrated the MLP combination effect, such as increasing *X* with *θ*_1_ and *t* factors on *b*_max_ (maintaining other MLPs at their optimal values) would increase *b*_max_. Since elevating *X* value is desired within mechanisms. Regarding the combined impact of *θ*_1_ at 45° with increasing *t* on *b*_max_ (refer to Figures 6(b) and 6(l)) is very important to limit either *t* or *θ*_1_ for the ideal mechanism.

### 4.4. Significance of Individual and Interaction Level of MLPs on *ѵ*

The variation of stiffness coefficient *ѵ* was found to be highly significant with MLPs such as *θ*_1_, followed by *t*, as their values maintain required stiffness in more than one direction since they are bicompatible mechanisms (depicted in Figure 5(c) of Pareto diagram). Normal data distribution of ERMs for *v*, observed to be above/below the line (as shown in Figure 5(d)), represents a good agreement between ERM and theoretical analysis. The impact of individual MLPs on *v* are depicted in Figure 7(a). Low values of *θ*_1_ and *t* and higher *F*-values attain maximum *v* when considering individually, thus fulfilling PRBM requirements. However, ∆ and *X* have the least impact on *v*, as they are the displacement results of other MLPs. The combined impact of MLPs (such as *F* medium-level value with every level of ∆, *X*, *θ*_1_, and *t*) provided the maximum *v* are as shown in Figures 7(b)to 7(f), suggesting *F* is insignificant in combination with other MLPs. Interactivity levels for MLPs (such as least ∆ value with increasing *X* and the medium value of *θ*_1_ and *t*) yield higher stiffness coefficients since *X* is adjustable in PRBM and has to be greater than ∆ (displayed in Figures 7(b) and 7(g)–7(i), respectively).

Similarly, combinatory levels of MLPs (such as least value of *θ*_1_ with increasing level of *X* with decreasing levels of *θ*_1_, and vice versa with *t*) yield maximum *v*. Since higher *X* cannot be obtained with thick links, loosening link stiffness and raising link 1 angle increase redundancy (plotted in surface responses Figures 7(b) and 7(j)–7(k)).  Figure 7(b) depicts combined impact levels for MLPs (such as least level of *θ*_1_ with any level of *t*) yielded maximum *v*, indicating that as long as *θ*_1_ and link 1 angle is minimum, links maintain their differing positions in such a manner as not to undergo buckling, in order to maintain stiffness.

### 4.5. Multiresponse GA-PSO of BCMs with MLPs

Multiple optimizing methods currently available for process responses only provide a single combination of optimized input parameter levels, which is not sufficient for manufacturers. Consequently, many possible sets of optimized input MLPs can easily be obtained by PSO for attaining a minimum of 90% of “*b*_max_” and 10% of “*v*” of the theoretical results. This would be very useful in presenting a BCCS with minimum actuation force and *X* > ∆, among other benefits. ERMs obtained from ANOVA of RS methodology have been characterized as the FFs. FFs of “*b*_max_ and *v*” from ERMs were to be modified in the standard form of the optimization model, as described in the following equations[20]:

(34) $$\begin{array}{c} F\left(1\right)=-0.1*\left(31.7+68*F-0.88*\Delta +0.58*X-0.25*\theta_{i}-5.2*t-10*F*F+0.0161*\Delta *\Delta +0.005*X*X-0.008*\theta_{i}*\theta_{i}-0.278*t*t-0.36*F*\Delta \right.\\ \left.+0.004*F*X-0.235*F*\theta_{i}-1.28*F*t-0.0384*\Delta *X+0.0358*\Delta *\theta_{i}+0.061*\Delta *t-0.0146*X*\theta_{i}+0.136*X*t-0.0178*\theta_{i}*t\right), \end{array}$$

(35) $$\begin{array}{c} F\left(2\right)=-0.9*\left(35.9-24.8*F-0.161*\Delta +1.042*X-3.155*\theta_{i}-\;0.48*t+6.59*F*F+0.0003*\Delta *\Delta -0.0196*X*X+0.03537*\theta_{i}*\theta_{i}+0.125*t*t-0.367*F*\Delta \right.\\ \left.+0.253*F*X+0.164*F*\theta_{i}-0.013*F*t+0.0165*\Delta *X-0.02202*\Delta *\theta_{i}-0.0016*\Delta *t+0.03954*X*\theta_{i}-0.0306*X*t+0.007*\theta_{i}*t\right). \end{array}$$

As both FFs are to be minimized, the “–” sign of both the functions *F*(1) and *F*(2) are to be multiplied for changing to minimization condition. The MLPs with higher and lower limits/bounds are provided to sort out all MLPs within a range, which are identified with “*b*_max_ and *v*” together. The possible MLP range is provided in Table 6.

GA employs mutation technique to prolong solution converging for Pareto front, obtained from PSO, to attain high-accuracy FF levels for the optimizing model [32]. Two outputs in the form of FFs were executed by the GA-PSO method through MATLAB's optimization toolbox. It produced several optimized-level combinations of MLPs, for an initial generation of 100 using multiple settings for standard values and Pareto-frontal diagrams to exhibit the best-global-optimized solutions (BGOS, shown in Figure 8). Corresponding values for BGOS are given in Table 7. Out of these 35 BGOS, 16 would fit best to meet the condition of *X* > ∆, minimum *F* and high *v*, to attain a successfully working mechanism that would not undergo buckling of linkages (provided in Table 8).

## 5. Conclusion

PRBM was theoretically constructed to develop bicompatible fixed-pinned beam and pinned-pinned beam mechanisms. Five MLPs (*F*, *X*, ∆, *θ*_1_, and *t*) and two outputs (maximum vertical footprint, *b*_max_, and the stiffness coefficient, *v*) were selected to obtain multiple potential mechanisms with conditions such as *X* > ∆, 90% *b*_max_, and 10% of *ѵ*, from theoretical results, along with minimal *F*/*θ*_1_. Presently, the available standard optimization techniques can provide only one set of optimized MLPs. However, GA-PSO presented a vast degree of information on all possible sets of optimized levels for MLP combinations. Initially, FFs are to be described as optimization models, requiring mathematical models of previously conducted theoretical studies. FFs utilize ERMs generated from the ANOVA of RSM for *b*_max_ and *v*, following checking of their competence and fitness with theoretical results. Using surface response 3D graphs, ERMs' individual factor levels/interaction levels of MLPs were studied, in order to understand the impact of MLP levels on outputs. Validation of these ERMs was carried out to check the good fit with theoretical results. GA-PSO analysis produced a large number of BGOS results at increased accuracy for a range of defined MLPs. Pareto-frontal diagram exhibited converged BGOS results during each generation, for two outputs. Stemming from such BGOS, at least 50% satisfy conditions prescribed with optimized MLP levels. Hence, GA-PSO proved to be highly practical in terms of producing large volumes of information to be utilized as a reference guide for designers.

GA-PSO can also be applied to other possible BCMs, can be compared with the present PRBM model, and consequently serves as a practical blueprint for a potential reference guide regarding such mechanisms.

## Figures and Tables

**Figure 1:** (a) The bistable compliant mechanism and (b) PRBM replacement of the bistable compliant mechanism.

**Figure 2:** Dimensional and forces analysis.

**Figure 3:** Steps involved in GA-PSO.

**Figure 4:** Deviation of RSM predicted values with theoretical model results for (a) *b*_max_ and (b) *v*.

**Figure 5:** Pareto diagram for (a) *b*_max_ and (c) *v* and normal probability distribution of residuals for (b) *b*_max_ and (d) *v*.

**Figure 6:** (a) Main effect of and (b–l) interaction effect of *F*, ∆, *X*, *θ*_1_, and *t* on *b*_max_.

**Figure 7:** (a) Main effect of and (b–l) interaction effect of *F*, ∆, *X*, *θ*_1_, and *t* on *v*.

**Figure 8:** Pareto front optimal solution plot.

**Table 1:** The constant coefficients for the fixed-pinned and pinned-pinned PRBMs, adopted from [1, 3].

	Γ	*ρ*	*K*Θ
Fixed-pined PRBM	0.85	0.85	2.65

**Table 2:** Operating factors [33].

Variables/parameters	Units	Values
*F*, maximum force	N	0.5, 1, 1.5, 2
Δ, CM maximum linear deflection	mm	20, 30, 40, 50, 60
*X*, CM maximum horizontal distance	mm	30, 40,50, 60,70
*θ*_1_, *L*_1_ initial angle	deg	20, 30, 40, 50, 60, 70
*t*, CM material thickness	mm	3, 6, 12

**Table 3:** CM analysis results, as per L27 orthogonal array.

No.	*F*	Δ	*X*	*θ*_1_	*t*	*L*_1_	*L*_2_	*θ*_2*i*_	*b*_max_	*ѵ*
1	0.5	20	30	20	3	21.28356	12.3689	36.05239	8.7	35
2	0.5	20	40	30	6	34.64102	20	60	19.8	30
3	0.5	20	50	40	12	52.21629	35.02201	73.40919	35	0.000001
4	0.5	30	60	50	6	70.00757	55.68716	74.3737	55.2	0.000001
5	0.5	30	70	60	12	110	96.43651	81.05172	96.25	0.000001
6	0.5	30	40	70	3	73.09511	70.30573	77.68103	70	0.000001
7	0.5	40	50	30	12	34.64102	26.45751	40.89339	22.95	10
8	1	40	60	40	3	52.21629	39.07098	59.21027	36.48	25
9	1	40	70	50	6	77.78619	62.85453	71.4462	62.23	23
10	1	50	50	60	12	50	50	60	46.8	6
11	1	50	60	70	3	102.3332	99.35831	75.42692	97.74	6
12	1	50	70	20	6	47.888	29.88746	33.23067	20.51	25
13	1	60	60	40	3	39.16222	39.16222	40	27.48	20
14	1	60	70	50	6	62.22895	56.32444	57.81678	52.22	12
15	1.5	60	70	60	12	80	75.49834	66.58678	74.76	6
16	1.5	20	30	70	6	58.47609	55.85206	79.6859	55.5	0.000001
17	1.5	20	40	20	12	31.92533	14.80631	47.51574	14.64	25
18	1.5	20	50	30	3	46.18802	25.16611	66.58678	24.75	70
19	1.5	30	60	50	6	70.00757	55.68716	74.3737	55.26	30
20	1.5	30	70	60	12	110	96.43651	81.05172	101.5	0.000001
21	1.5	30	40	70	3	73.09511	70.30573	77.68103	68.64	10
22	2	40	50	20	12	31.92533	22.78655	28.63257	13.35	25
23	2	40	60	30	3	46.18802	30.5505	49.10661	25.44	40
24	2	40	70	40	6	65.27036	46.47817	64.5128	45.08	30
25	2	50	50	60	3	50	50	60	44.55	25
26	2	50	60	70	6	102.3332	99.35831	75.42692	97.74	6
27	2	50	70	50	12	70.00757	59.16976	65.00665	58.1	13
								Important (40%), **maximized**	Very important (90%), **minimized**	Very important (10%), **minimized**

**Table 4:** Analysis of variance for responses *b*_max_ and *v*.

Source	*b*_max_					*v*				
	DF	Adj. SS	Adj. MS	*F*-value	*P*-value	DF	Adj. SS	Adj. MS	*F*-value	*P*-value
Model	20	19998.5	999.93	170.28	≤0.001	20	6542.72	327.136	5.74	0.019
Linear	5	5793.5	1158.70	197.32	≤0.001	5	1582.78	316.556	5.55	0.030
*F*	1	32.0	32.02	5.45	0.058	1	234.74	234.741	4.12	0.089
Δ	1	188.1	188.09	32.03	0.001	1	3.69	3.689	0.06	0.808
*X*	1	826.3	826.28	140.71	≤0.001	1	2.61	2.613	0.05	0.838
*θ*_1_	1	3165.6	3165.59	539.08	≤0.001	1	807.97	807.965	14.17	0.009
*T*	1	1.0	1.04	0.18	0.688	1	717.46	717.457	12.59	0.012
Square	5	957.8	191.56	32.62	≤0.001	5	172.69	34.539	0.61	0.701
*F∗F*	1	8.4	8.37	1.43	0.278	1	19.41	19.414	0.34	0.581
Δ*∗*Δ	1	0.0	0.00	0.00	0.982	1	7.68	7.684	0.13	0.726
*X∗X*	1	11.5	11.49	1.96	0.211	1	0.76	0.762	0.01	0.912
*θ*_*i*_*∗θ*_*i*_	1	625.0	625.03	106.44	≤0.001	1	32.09	32.089	0.56	0.481
*t∗t*	1	3.4	3.38	0.57	0.477	1	16.71	16.705	0.29	0.608
Two-way interaction	10	695.8	69.58	11.85	0.003	10	944.44	94.444	1.66	0.277
*F∗*Δ	1	11.5	11.49	1.96	0.211	1	11.00	10.999	0.19	0.676
*F∗X*	1	23.1	23.07	3.93	0.095	1	0.00	0.004	0.00	0.993
*F∗θ*_1_	1	14.4	14.45	2.46	0.168	1	29.63	29.629	0.52	0.498
*F∗t*	1	0.0	0.00	0.00	0.978	1	50.38	50.376	0.88	0.383
Δ*∗X*	1	5.2	5.25	0.89	0.381	1	28.45	28.453	0.50	0.506
Δ*∗θ*_1_	1	28.6	28.64	4.88	0.069	1	75.61	75.611	1.33	0.293
Δ*∗t*	1	0.0	0.01	0.00	0.968	1	14.81	14.813	0.26	0.628
*X∗θ*_1_	1	157.5	157.46	26.82	0.002	1	21.53	21.534	0.38	0.561
*X∗t*	1	1.3	1.27	0.22	0.658	1	25.14	25.142	0.44	0.531
*θ*_*i*_*∗t*	1	0.8	0.82	0.14	0.722	1	5.33	5.333	0.09	0.770
Error	6	35.2	5.87			6	342.02	57.003		
Total	26	20,033.8				26	6,884.74			
**R** ^**2**^		99.82%					95.02%			
**R** ^**2**^ **(adjusted)**		99.24%					92.24%			

**Table 5:** Authentication of stochastic model results for *b*_max_ and *v*.

No.	Input attributes					*b*_max_			*V*		
	*F*	Δ	*v*	*θ*_1_	*T*	Predicted	Numerical	Deviation	Predicted	Numerical	Deviation
1	0.5	20	30	20	3	10.532	9.7	0.832	37.18	36	1.18
2	0.5	20	40	30	6	16.1415	17.8	1.6585	26.443	28	.557
3	0.5	20	50	40	12	36.2165	35	1.2165	0.0164	0.000001	0.0163999
4	0.5	30	60	50	6	57.0745	55.2	1.8745	0.0767	0.000001	0.0767
5	0.5	30	70	60	12	95.7935	96.25	0.4565	0.068	0.000001	0.068
6	0.5	30	40	70	3	70.255	70	0.255	0.485	0.000001	0.485
7	0.5	40	50	30	12	22.3555	22.95	0.5945	8.555	10	1.445
8	1	40	60	40	3	35.192	36.48	1.288	24.502	25	0.498
9	1	40	70	50	6	61.491	62.23	0.739	17.502	18	0.498
10	1	50	50	60	12	47.276	46.8	0.476	6.942	6	0.942
11	1	50	60	70	3	96.989	97.74	0.751	4.57	5	0.43
12	1	50	70	20	6	21.114	20.51	0.604	25.786	25	0.786
13	1	60	60	40	3	27.32	27.48	0.16	18.122	20	1.878
14	1	60	70	50	6	52.419	52.22	0.199	14.262	13	1.262
15	1.5	60	70	60	12	74.4605	74.76	0.2995	8.682	6	2.682
16	1.5	20	30	70	6	54.9545	55.5	0.5455	0.039	0.000001	0.039
17	1.5	20	40	20	12	15.5235	14.64	0.8835	27.526	25	2.526
18	1.5	20	50	30	3	24.224	24.75	0.526	65.541	70	4.459
19	1.5	30	60	50	6	57.7465	56.26	1.4865	28.777	30	1.223
20	1.5	30	70	60	12	100.5575	101.5	0.9425	4.052	0.000001	4.051999
21	1.5	30	40	70	3	69.186	68.64	0.546	15.585	10	5.585
22	2	40	50	20	12	12.752	13.35	0.598	24.456	25	0.544
23	2	40	60	30	3	25.568	25.44	0.128	42.876	40	2.876
24	2	40	70	40	6	44.76	45.08	0.32	33.32	30	3.32
25	2	50	50	60	3	44.619	44.55	0.069	26.014	25	1.014
26	2	50	60	70	6	97.809	97.74	0.069	3.626	6	2.374
27	2	50	70	50	12	58.609	58.1	0.509	8.618	10	1.382

**Table 6:** Higher/lower limits for MLPs.

MLPs	Lower bound	Upper bound
*F*, maximum force	0.5	2
Δ, the mechanism's maximum linear deflection	20	60
*X*, the maximum horizontal footprint	30	70
*θ*_1_, the initial angle of segment 1	20	70
*t*, the material thickness	3	12

**Table 7:** BGOS results from GA-PSO analysis.

No.	*F*	∆	*X*	*θ*_1_	*T*	*b*_max_	*V*
1	1.9998	59.9914	30.00	41.7493	4.92698	41.823	5.955
2	1.9237	43.0343	30.382	48.6654	11.907	11.2031	0.032
3	0.5001	20.904	31.614	69.995	11.996	59.2433	5.688
4	1.977	58.409	30.2795	44.285	11.893	33.2414	1.9886
5	0.5985	22.714	31.026	56.947	11.982	28.607	3.60
6	1.883	37.7573	30.451	50.562	11.958	2.3198	0.726
7	0.8138	23.428	31.251	47.0983	11.965	13.9895	2.03
8	1.9061	44.1491	30.293	46.0847	11.722	15.0369	0.404
9	1.77996	41.7163	31.037	50.5222	11.9644	6.15796	0.175
10	0.8601	23.9132	30.637	55.96	11.959	23.34898	2.92
11	0.67752	21.6944	30.837	63.89	11.967	41.5582	4.454
12	1.12264	33.994	30.552	49.90	11.922	3.22183	0.903
13	1.9985	59.80	30.037	42.06	8.2111	40.261	4.486
14	0.54854	21.4851	31.5014	63.84	11.9748	43.948	4.662
15	1.33695	24.9752	30.541	57.41	11.7094	22.759	2.352
16	1.6883	37.2185	30.455	53.49	11.9291	1.527	0.832
17	1.98075	59.6126	30.150	43.345	10.7384	36.904	2.971
18	0.5378	22.2681	31.1297	66.3756	11.986	47.72	4.933
19	1.2685	29.1801	30.6187	48.6358	11.9111	6.52	1.188
20	1.0924	21.3485	31.1169	49.832	11.9169	17.56	2.068
21	1.9726	54.6815	30.3481	45.144	11.9149	28.1896	1.453
22	1.9744	50.3403	30.3173	43.003	11.8225	23.962	1.027
23	1.9759	56.9533	30.31561	44.445	11.8585	31.391	1.809
24	1.9997	59.862	30.008	41.812	6.01313	41.517	5.529
25	1.9981	59.743	30.020	42.0933	7.00447	40.966	5.087
26	0.5174	21.811	31.25923	58.888	11.992	33.8772	4.092
27	1.1291	28.3411	30.7832	50.6212	11.961	10.4791	1.583
28	0.556	22.25	31.2735	53.849	11.9693	25.165	3.356
29	1.995	59.7552	30.041	42.383	8.656	39.7974	4.248
30	1.5072	26.9654	30.5069	56.1037	11.951	18.597	2.175
31	1.9809	59.636	30.1347	42.631	9.9818	38.006	3.461
32	0.50046	20.989	31.5538	69.508	11.987	57.778	5.602
33	0.58476	23.5454	31.5981	69.745	11.980	54.781	5.0554
34	0.55682	22.295	31.212	58.564	11.972	32.389	3.8997
35	1.91224	47.794	30.3511	45.3443	11.8143	19.667	0.7571

**Table 8:** BGOS results satisfying designer requirements.

No.	*F*	∆	*X*	*θ*_1_	*T*	*b*_max_	*V*
1	0.5001	20.904	31.614	69.995	11.996	59.2433	5.688
2	0.5985	22.714	31.026	56.947	11.982	28.607	3.60
3	0.8138	23.428	31.251	47.0983	11.965	13.9895	2.03
4	0.8601	23.9132	30.637	55.96	11.959	23.34898	2.92
5	0.67752	21.6944	30.837	63.89	11.967	41.5582	4.454
6	0.54854	21.4851	31.5014	63.84	11.9748	43.948	4.662
7	0.5378	22.2681	31.1297	66.3756	11.986	47.72	4.933
8	1.2685	29.1801	30.6187	48.6358	11.9111	6.52	1.188
9	1.0924	21.3485	31.1169	49.832	11.9169	17.56	2.068
10	0.5174	21.811	31.25923	58.888	11.992	33.8772	4.092
11	1.1291	28.3411	30.7832	50.6212	11.961	10.4791	1.583
12	0.556	22.25	31.2735	53.849	11.9693	25.165	3.356
13	1.5072	26.9654	30.5069	56.1037	11.951	18.597	2.175
14	0.50046	20.989	31.5538	69.508	11.987	57.778	5.602
15	0.58476	23.5454	31.5981	69.745	11.980	54.781	5.0554
16	0.55682	22.295	31.212	58.564	11.972	32.389	3.8997

## Data Availability

The data used to support the findings of this study are available from the corresponding author upon request.
